# Reduced miR-125a-5p level in non-small-cell lung cancer is associated with tumour progression

**DOI:** 10.1098/rsob.180118

**Published:** 2018-10-10

**Authors:** Hongxu Liu, Yegang Ma, Changhao Liu, Pengfei Li, Tao Yu

**Affiliations:** 1 Department of Thoracic Surgery, Cancer Hospital of China Medical University, Shenyang 110042, Liaoning Province, People's Republic of China; 2 Department of Medical Imaging, Cancer Hospital of China Medical University, Shenyang 110042, Liaoning Province, People's Republic of China; 3 Department of Thoracic Surgery, Liaoning Cancer Hospital and Institute, Shenyang 110042, Liaoning Province, People's Republic of China; 4 Department of Medical Imaging, Liaoning Cancer Hospital and Institute, Shenyang 110042, Liaoning Province, People's Republic of China

**Keywords:** miR-125a-5p, non-small-cell lung cancer, Suv39H1

## Abstract

Emerging evidence suggests that microRNAs (miRNAs) serve an important role in tumourigenesis and development. Although the low expression of miR-125a-5p in non-small-cell lung cancer (NSCLC) has been reported, the underlying mechanism remains unknown. In the current study, the low expression of miR-125a-5p in NSCLC was verified in paired cancer tissues and adjacent non-tumour tissues. Furthermore, the CpG island in the miR-125a-5p region was hypermethylated in the tumour tissues, and the hypermethylation was negatively correlated with miR-125a-5p expression. Target gene screening showed that the histone methyltransferase Suv39H1 was one of the potential target genes. *In vitro* studies showed that miR-125a-5p could directly suppress Suv39H1 expression and decrease the H3K9me3 levels. On the other hand, Suv39H1 could induce demethylation of miR-125a-5p, resulting in re-activation of miR-125a-5p. What is more, overexpessing miR-125a-5p could also self-activate the silenced miR-125a-5p in NSCLC cells, which suppressed cell migration, invasion and proliferation *in vitro* and inhibited cancer progression *in vivo*. Thus, we found that the epigenetic silenced miR-125a-5p could be self-activated through targeting Suv39H1 in NSCLC, suggesting that miR-125a-5p might not only have the potential prognostic value as a tumour biomarker but also be a potential therapeutic target in NSCLC.

## 1. Introduction

Lung cancer is currently the most common cause of tumour-related mortality in the world [1–3]. There are two main subtypes of lung cancer, small-cell lung carcinoma and non-small-cell lung carcinoma (NSCLC), accounting for 15% and 85% of all lung cancer, respectively [1–4]. Clinically, NSCLC is frequently diagnosed at advanced stages of disease [4]. Over half of patients diagnosed with lung cancer die within 1 year of diagnosis and the 5-year survivals are around 17.8% [1–3]. Moreover, NSCLC patients are relatively insensitive to chemo- and radio-therapy [4]. Despite advances in early detection, radical surgical resection and multimodal therapeutic modalities over the recent decades, the long-term survival remains poor due to the high rate of recurrence and metastasis [1].

Therefore, there is an urgent need to identify novel biomarkers that will help select the patients with a high chance of lung cancer recurrence and uncover the underlying mechanisms that would provide better targets for NSCLC treatment. An increasing amount of evidence shows that various microRNAs (miRNAs), a novel class of small (20–24 nucleotides) non-coding regulatory RNAs, are related in terms of tumour formation, development, progression and the responses to the treatment [5–7], including lung cancer [8–10]. Among all the dysregulated miRNAs, miR-125a-5p is one of the most downregulated miRNAs in NSCLC [8–10].

A number of studies have shown that the miRNA-125a-5p is an important tumour suppressor and its expression is reduced in many types of human cancer, including laryngeal cancer [11], juvenile angiofibromas [12], colorectal cancer [13], breast cancer [14,15], lung cancer [8–10], cervical carcinomas [16], prostate and pancreatic cancers [17]. miRNA-125a-5p has been demonstrated as an independent prognostic factor in gastric cancer and inhibiting gastric cancer development [18], through targeting oncogenes such as vascular endothelial growth factor A [19] and E2F transcription factor 3 [20]. Over-expressing miR-125a-5p could inhibit the cancer proliferation and migration [21,22].

However, the underlying mechanism of the low expression of miR-125a-5p in NSCLC remains unknown. It has been demonstrated that some epigenetic modulators could modulate the miR-125-5p expression, such as HDACs (histone deacetylases) [14,23], or be modulated by miR-125-5p, such as Sirtuins [24]. Furthermore, the putative promoter regions in the miR-125a-5p are embedded in CpG islands, and are hypermethylated in glioma cells [25]. Considering the above findings, we wanted to test the expression and methylation status of miR-125a-5p in NSCLC tissues and adjacent non-tumour tissues, and then evaluate whether DNA methylation participates in regulating miR-125a-5p expression in human NSCLC.

In the present study, it was confirmed that miR-125a-5p expression was reduced in most NSCLC tissues compared with the adjacent non-tumour tissues. DNA methylation analysis showed the miR-125a-5p promoter was highly methylated and negatively associated with its expression. Target gene screening and validation showed that the histone methyltransferase Suv39H1 is the miR-125a-5p target gene, which was also involved in the epigenetic silencing of the miR-125a-5p. Overexpressing miR-125a-5p could self-activate the silenced miR-125a-5p in NSCLC cells, resulting in cancer suppression *in vitro* and *in vivo*. The data here show that miR-125a-5p might not only have potential prognostic values as a tumour biomarker but also be a potential therapeutic target in NSCLC.

## 2. Material and methods

### 2.1. Patients

A total of 384 patients histologically verified NSCLC at the Cancer Hospital of China Medical University, Liaoning Cancer Hospital and Institute, between 2005 and 2016 were enrolled in this study. The median age of the patients was 55.6 years (range 29–76 years). None of them received any pre-operative anti-cancer treatment prior to sample collection. This study was approved by the local ethics committee of the Cancer Hospital of China Medical University, Liaoning Cancer Hospital and Institute, and written informed consent was obtained from each patient. All 384 specimens were reevaluated with respect to their histological types, differentiation status, smoking status and tumour TNM stages. Tumour stages were determined by TNM classification according to the 2002 International Union against Cancer guidelines. The histological diagnosis and grade of differentiation of the tumours were defined by evaluation of the haematoxylin and eosin-stained tissue sections, according to the World Health Organization guidelines of classification (2004). Tissues were collected within 1 h after surgery. Every patient specimen included two matched pairs, namely NSCLC tissues and adjacent normal lung tissues (greater than or equal to 5 cm away from the tumour). For each specimen, half were immediately flash-frozen in liquid nitrogen and then frozen at −80°C until RNA and DNA extraction was performed, the remainder was fixed with formalin for immunohistochemistry.

### 2.2. RNA isolation and RT–qPCR

Total RNA from tissues or cultured cells were isolated using TRIzol reagent (Thermo Fisher Scientific, Rockford, IL, USA) according to the manufacturer's protocol. RNA concentration was measured using NanoDrop ND-1000 (Thermo Fisher Scientific) and the quality was assessed using electrophoresis with 1.5% denaturing agarose gels. TaqMan probe-based qPCR was performed using a commercial kit (Applied Biosystems, Thermo Fisher Scientific) according to the manufacturer's protocol. Reverse transcription was performed using a miR-125a-5p specific primer and ABI's TaqMan MicroRNA Reverse Transcription kit (Applied Biosystems, Thermo Fisher Scientific). miR-125a-5p expression level was detected using a Taqman MicroRNA assay (Applied Biosystems, Thermo Fisher Scientific) with the Applied Biosystems 7900HT Sequence Detection system. U6 was used as the internal control. The RT–qPCR thermocycling conditions were as follows: 94°C for 30 s (initial denaturation), 94°C for 5 s (denaturation) and 55°C for 30 s (annealing), for 40 cycles. The following primers were used: miR-125a-5p forward, 5'-GGTAAGTCACGCGGT-3′ and reverse, 5'-CAGTGCGTCTCGTGGAGT-3′; U6 forward, 5'-CTGGTTAGTACTTGGACGGGAGAC-3′ and reverse, 5'-GTG CAGGGTCCGAGGT-3′. Subsequently, the 2^−ΔΔ^Ct method was used to quantify the expression level of the miRNA relative to U6.

### 2.3. DNA extraction and methylation analysis

Genomic DNA was isolated from tissues or cultured cells by using the Universal Genomic DNA Extraction Kit v. 3.0 (Takara) in accordance with the manufacturer's instructions. The quality and integrity of DNA were checked by electrophoresis on 1% agarose gel, quantified spectrophotometrically. Bisulfite modification of DNA was produced by using the EpiTect Bisulfite Kit (Qiagen) according to the manufacturer's recommendations. In brief, the DNA (1 µg) was denatured using NaOH and subsequently modified by sodium bisulfite. Then, the mixture was desulfonated, and DNA was purified on silica-membrane columns. The bisulfite-treated miR-125a-5p promoter regions containing CpG sites was amplified and subcloned into a pGEM T-Easy vector (Promega) after gel purification. There were 23 CpG sites in total were analysed, starting from −680 to −374 bp upstream of the miR-125a-5p sequences. The primer sequences used for miR-125a-5p promoter analysis were: forward primer 5′-GGATTTTTGGGTTTTGGTATTTATT-3′ and reverse primer 5′-AAATATCCTCCTCAACTATACAACCTC-3′. The resulting products were next transformed into JM109 competent cells. Methylation states of each CpG site were analysed by randomly sequencing 10 clones. The methylation level for each sample was calculated as the percentage of methylated CpG dinucleotides from the total number of CpG dinucleotides.

### 2.4. Cell culture

The A549 and SK-MES-1 human NSCLC cell lines were obtained from the American Type Culture Collection (ATCC; Rockville, MD, USA). The cell line HEK293T was purchased from China Center for type culture collection in Wuhan. All cells were cultured in DMEM (GIBCO, Shanghai, China) supplemented with 10% FBS. miRNA was transfected at 30 nM (final concentration) using Lipofectamine RNAiMAX (Thermo Fisher Scientific) according to the manufacturer's instructions.

### 2.5. Luciferase reporter assay

The 3'-UTR of human Suv39H1 containing the potential miR-125a-5p was amplified by high-fidelity PCR. Then the amplified sequence was cloned into the XbaI site of the pGL3 control vector (Promega). The mutated putative miR-125a-5p binding site in the 3'-UTR of Suv39H1 was generated using the QuickChange Site-directed Mutagenesis kit (Stratagene) according to the manufacturer's protocol. The day before transfection, HEK293T cells were seeded in 24-well plates (5 × 10^4^ cells well^−1^), then we transfected 500 ng Suv39H1 3'-UTR-pGL3 and 30 nM (final concentration) miR-125a-5p mimics or control miRNA mimics (Ambion) into the cells with Lipofectamine 2000. Forty-eight hours after transfection, luciferase activity was determined using dual-luciferase reporter assay system (Promega) according to the manufacturer's protocol.

### 2.6. Western blotting

Total protein from tumour tissues or cultured cells were lysed in RIPA buffer with protease inhibitor (Beyotime, Shanghai, China). The protein was quantified using a BCA assay kit (Beyotime). A total of 20 µg of total protein were separated by 10% SDS–PAGE, transferred onto polyvinylidene fluoride membranes, and then reacted with primary antibodies against Suv39H1, H3K9me3 and β-actin (Abcam). After being extensively washed with PBS containing 0.1% Triton X-100, the membranes were incubated with alkaline phosphatase-conjugated goat anti-rabbit antibody for 30 min at room temperature. The bands were visualized using one-step TM NBT/BCIP reagents (Thermo Fisher Scientific) and detected by an Alpha Imager (Alpha Innotech, San Leandro, CA, USA).

### 2.7. Cell viability assay

Cell viability was evaluated using CCK-8 (Beyotime) according to the manufacturer's instructions. Briefly, cells were seeded into 96-well plates at 5 × 10^3^ cells per well and cultured for indicated time points. Ten microlitres of CCK-8 solution were added into the culture medium in each well. After 1 h incubation, optical density values were read using a microplate reader (Bio-Tek Company, Winooski, VT, USA) at the 450 nm wavelength. Each time point was repeated in three wells and the experiment was independently performed three times.

### 2.8. Cell apoptosis assay

Cell apoptosis was evaluated by flow cytometry using an Annexin V-FITC Apoptosis Detection Kit (KeyGen Biotech Co. Roche, Nanjing, China). Briefly, cells were seeded into 24-well plates at 1 × 10^5^ cells per well and cultured for 48 h. Then the cells were detached by trypsinization, washed twice in PBS (2000 r.p.m., 5 min; Allegra X-12R centrifuge; Beckman Coulter, USA), and resuspended in 500 µl binding buffer. A volume of 5 µl Annexin V-FITC and 5 µl propidium iodide was added and mixed gently, and the cells were stained in the dark for 10 min at room temperature. The cells were analysed immediately by flow cytometry (BD FACSCalibur, BD Bioscience, San Diego, CA, USA) and analysed using Flowjo software (FlowJo, Ashland, OR, USA). The experiment was repeated three times.

### 2.9. Cell migration assay

The migration of cells was detected by wound healing assay. Cells were cultured in 6-well plates. When the cells grew to 80–90% confluence, a wound in a line across the well was made by a plastic pipette tip. The area of cell-free wound was recorded 24 h after incubation with rhIL-35 protein using an inverted microscope and analysed by the NIH Image 1.55 software. Percentage wound healing was calculated as 100 × (1 − the remaining cell-free area/the area of the initial wound). All tests were performed in triplicate.

### 2.10. Transwell invasion assay

Invasive ability of cells was determined within a transwell system. A total of 6.0 × 10^4^ cells were seeded onto the upper surface of the transwell membrane and cultured at 37°C in 5% CO_2_ for 24, 48 and 72 h. The number of cells that migrated to the lower surface of the membrane was counted under a microscope (200×).

### 2.11. Lentivirus preparation

The miR-125a-5p was cloned into lentiviral pLKO.1-puro vector, and the empty vector as negative control. Lentiviruses were prepared using HEK293T cells according to the manufacturer's instructions. A549 cells were incubated with lentivirus and 4 µg ml^−1^ polybrene (AmericanBio) for 24 h.

### 2.12. Animal study

Six- to eight-week-old nude mice (Charles River Laboratories, Beijing, China) were housed in specific pathogen-free conditions. The study was approved by the Research Ethics Committee of Cancer Hospital of China Medical University, Liaoning Cancer Hospital and Institute. Mice were housed in the pathogen-free region and monitored daily during the experiments and the mice would be sacrificed when the weight loss is more than 20%. For evaluation of the tumour growth *in vivo*, 5 × 10^6^ A549 cells were suspended in 200 µl PBS and injected subcutaneously into the dorsal scapula region of the mice. Four weeks later, the tumour size was measured with fine digital calipers and calculated by the following formula: tumour volume = 0.5 × width^2^ × length.

### 2.13. Statistical analysis

Data were expressed as mean (±s.e.) and analysed by SPSS software (SPSS Standard v. 13.0, SPSS Inc., USA). Differences between variables were assessed by the *χ*^2^ test. Survival analysis was calculated by the Kaplan–Meier analysis. A log-rank test was used to compare different survival curves. A Cox proportional hazards model was used to calculate univariate and multivariate hazard ratios for the variables. Unpaired Student's *t*-test and one-way ANOVA were used as appropriate to assess the statistical significant of difference. *p*-values under 0.05 were considered statistically significant.

## 3. Results

### 3.1. Decreased miR-125a-5p expression in human non-small-cell lung cancer

A total of 384 cases with NSCLC were followed (table 1). All these patients had received no pre-operation chemotherapy. They were given the same radical operation and underwent the same adjuvant chemotherapy after the surgery. We first analysed the miR-125a-5p expression in 384 NSCLC specimens. The data showed that the miR-125a-5p level reduced significantly in NSCLC comparing with its paired adjacent non-cancerous tissues (figure 1*a*). The downregulation of miR-125a-5p might be related to the cancer progression; thus, the samples were divided into two groups, the ‘high’ and ‘low’ groups, according to their relative expression levels of miR-125a-5p to internal control U6. The reduced miR-125a-5p level was associated with TNM stages (*p* < 0.01), AJCC stage (*p* = 0.008), differentiation (*p* = 0.002) and vascular invasion (*p* = 0.002; table 1)

**Figure 1.** Reduced miR-125a-5p is correlated with the poor prognosis of NSCLC. (*a*) miR-125a-5p levels in cancer tissues and adjacent normal tissues were determined by qPCR (*n* = 384). The middle line indicates median; bottom of box, 25th percentile; top of box, 75th percentile. *p < 0.05. (*b*) Kaplan–Meier survival curve of patients with high or low level of miR-125a-5p. (*c*) miR-125a-5p methylation levels in cancer tissues and adjacent normal tissues were determined (*n* = 384). The middle line indicates median; bottom of box, 25th percentile; top of box, 75th percentile. *p < 0.05. (*d*) Correlation between the mRNA level and the methylation level of miR-125a-5p.

**Table 1.** Association between clinicopathological features and miR-125a-5p expression. *p < 0.05 indicates a significant association among the variables.

		miR-125a-5p expression in tumour		
	*n*	high (*n* = 292, %)	low (*n* = 92, %)	*p*-value
age, years			0.393	
<65	170	34.0	45.0	
≥65	214	66.0	55.0	
gender				0.521
male	180	48.4	39.1	
female	204	51.6	60.9	
T stage				0.008*
T1	6	3.2	3.0	
T2	21	16.1	5.7	
T3	172	46.9	29.1	
T4	185	33.8	62.2	
N stage				0.005*
N0	94	67.7	40.7	
N1	158	25.7	34.7	
N2	132	6.6	24.6	
M stage				0.001*
M0	268	96.8	81.3	
M1	116	3.2	18.7	
AJCC stage				0.008*
I	72	17.7	7.2	
II	119	46.8	31.9	
III	125	32.2	42.0	
IV	68	3.3	18.9	
differentiation				0.002*
high	88	66.0	32.0	
moderate	168	27.4	41.0	
low	128	6.6	27.0	
vascular invasion				0.002*
yes	273	96.8	91.4	
no	111	3.2	8.6	

Patient follow-up was carried out for all patients who had undergone curative operations. The Kaplan–Meier curves with a log-rank test for overall survival (OS) and disease-free survival (DFS) was conducted to assess the predictive role of miR-125a-5p for distant metastasis. There was a significant difference between the high and low miR-125a-5p groups after the surgery (figure 1*b*). Patients with low miR-125a-5p expression subsequently developed more metastasis or local recurrence than those with high miR-125a-5p expression (*p* < 0.01). When compared with patients with high miR-125a-5p expression, the DFS rate was significantly lower in patients who had low expression of miR-125a-5p (figure 1*b*; log-rank test, *p* < 0.001). The Kaplan–Meier analysis also revealed that the miR-125a-5p expression was significantly relevant to OS of NSCLC patients (figure 1*b*; log-rank test, *p* < 0.001). Patients with low expression of miR-125a-5p had a significantly lower 5-year OS than those with high miR-125a-5p expression.

Univariate analysis showed that the NSCLC patients with low miR-125a-5p expression had a significantly lower DFS and OS than those with high miR-125a-5p levels (table 2). In multivariate analysis with clinicopathologic parameters, the low miR-125a-5p expression was found to be an independent prognostic marker to predict tumour recurrence (table 3).

**Table 2.** Univariate Cox proportional hazards model for DFS and OS. *p < 0.05 indicates a significant association among the variables. HR, hazard ratio.

	DFS			OS		
	HR	95% CI	*p*-value	HR	95% CI	*p*-value
age, years						
<65	—			—		
≥65	1.009	0.659–1.841	0.714	0.934	0.530–1.644	0.822
AJCC stage						
I	—			—		
II	1.108	0.305–4.027	0.877	0.667	0.201–2.215	0.518
III	6.823	2.097–22.199	0.001*	3.401	1.184–9.771	0.026*
IV	49.185	12.615–191.764	<0.001*	40.074	11.257–142.668	<0.001*
differentiation						
high	—			—		
moderate	1.315	0.750–2.306	0.341	1.458	0.764–2.780	0.273
low	3.577	1.885–6.786	<0.001*	4.358	2.140–8.872	<0.001*
vascular invasion						
yes	4.901	2.469–9.721	<0.001*	4.638	2.152–9.997	<0.001*
no	—			—		
miR-125a-5p						
high	—			—		
low	6.118	3.004–12.462	<0.001*	6.348	2.875–14.014	<0.001*

**Table 3.** Multivariate Cox proportional hazards model for DFS and OS. *p < 0.05 indicates a significant association among the variables. HR, hazard ratio.

	DFS			OS		
	HR	95% CI	*p*-value	HR	95% CI	*p-*value
miR-125a-5p level	2.796	1.919–4.161	<0.001*	2.659	1.711–4.223	<0.001*
T stage	1.701	1.129–2.541	0.008*	3.981	1.854–9.173	<0.001*
N stage	3.698	2.049–6.701	<0.001*	3.321	1.813–6.203	<0.001*
M stage	4.402	1.299–14.551	0.011*	8.001	2.403–26.815	<0.001*

It has been demonstrated that the epigenetic modulators could modulate the miR-125-5p expression [14,23,24], and its promoter is hypermethylated in glioma cells [25]. We analysed the miR-125a-5p methylation status in NSCLC and adjacent non-tumour tissues. We designed and validated bisulfate sequencing PCR for the promoter region of miR-125a-5p including 20 CpGs. Data showed that the miR-125a-5p was hypermethylated in NSCLC comparing with the adjacent non-cancer tissues (figure 1*c*). To further determine whether DNA methylation contributes to the silencing of miR-125a-5p in NSCLC, the correlation between the miR-125a-5p and its methylation level was analysed. And the methylation status was negatively correlated with its expression level (figure 1*d*).

Taken together, these results suggested that the epigenetic silenced miR-125a-5p might contribute to NSCLC development and the poor outcomes.

### 3.2. Suv39H1 is directly regulated by miR-125a-5p

To uncover the potential mechanism of the epigenetic silencing of miR-125a-5p in NSCLC cells, the potential targets of miR-125a-5p were screened by using prediction tools including miRanda, TargetScan and Pictar algorithms. Among the hundreds of targets that were predicted, the histone methyltransferase Suv39H1 was further studied. To obtain the direct evidence that Suv39H1 is a potential target of miR-125a-5p, we examined whether the predicted binding sites of miR-125a-5p in the 3′-UTR of Suv39H1 mRNA were responsible for its regulation (figure 2*a*). The 3'-UTR of Suv39H1 was cloned into the downstream of a luciferase reporter, and this vector was co-transfected with an miR-125a-5p mimic or its negative control into HEK293T cells. The luciferase activity of cells transfected with miR-125a-5p mimic was significantly reduced compared with the negative control (*p* < 0.05; figure 2*b*). Furthermore, deletion of the putative binding site clearly abrogated the repression of luciferase activity caused by miR-125a-5p over-expression (figure 2*b*).

**Figure 2.** Suv39H1 is the miR-125a-5p target gene. (*a*) The potential binding site of miR-125a-5p in the 3′UTR of Suv39H1. (*b*) Luciferase assay performed by over-expressing miR-125a-5p and the wild-type of Suv39H1 3′UTR (WT-3′UTR) or the 3′UTR without potential miR-125a-5p binding site (Mut-3′UTR). *n* = 3. *p < 0.05. (*c*) Suv39H1 levels in cancer tissues and adjacent normal tissues were determined by qPCR (*n* = 384). The middle line indicates median; bottom of box, 25th percentile; top of box, 75th percentile. *p < 0.05. (*d*) Over-expressing miR-125a-5p could suppress the Suv39H1 expression in NSCLC cell lines (A549 and SK-MES-1), determined by qPCR. *n* = 3. *p < 0.05. (*e*) Over-expressing miR-125a-5p could suppress the Suv39H1 expression in NSCLC cell lines (A549 and SK-MES-1), determined by western blot. NC: empty vector.

If the Suv39H1 is regulated by miR-125a-5p in NSCLC, the Suv39H1 expression level in NSCLC should be upregulated as the downregulation of miR-125a-5p. As expected, the mRNA level of Suv39H1 was upregulated in NSCLC comparing with the adjacent non-tumour tissues (figure 2*c*). After over-expressing miR-125a-5p, the mRNA and protein levels of Suv39H1 was suppressed significantly (figure 2*d,e*).

These data suggested that miR-125a-5p might inhibit the Suv39H1 expression through 3′-UTR in NSCLC, and affect the epigenetic status of the cancer cells.

### 3.3. Demethylation and activation of endogenous miR-125a-5p through exogenous over-expressing miR-125a-5p

Because Suv39H1 is a histone-lysine *N*-methyltransferase that specifically trimethylates Lys-9 of histone H3 (H3K9me3), we first determined whether over-expressing miR-125a-5p would affect the H3K9 trimethylation (H3K9me3) status through targeting Suv39H1. As expected, the whole genome H3K9me3 level was decreased after over-expressing miR-125a-5p (figure 3*a*). H3K9me3 is also tightly related to the DNA methylation. Thus, we then measured the miR-125a-5p methylation level after miR-125a-5p over-expression. Interestingly, the methylation level was decreased by over-expressing miR-125a-5p (figure 3*b*). Furthermore, the endogenous miR-125a-5p precursor was also upregulated (figure 3*c*). This upregulation and demethylation of miR-125a-5p were abolished when over-expressing miR-125a-5p and Suv39H1 together (figure 3*d–f*), indicating that miR-125a-5p could modulate its own methylation and expression through Suv39H1.

**Figure 3.** Demethylation and activation of endogenous miR-125a-5p through exogenous over-expressing miR-125a-5p. (*a*) Over-expressing miR-125a-5p could suppress the H3K9me3 level in NSCLC cell lines (A549 and SK-MES-1), determined by western blot. (*b*) Over-expressing miR-125a-5p could suppress the miR-125a-5p methylation levels in NSCLC cell lines (A549 and SK-MES-1). *n* = 3. *p < 0.05. (*c*) Over-expressing miR-125a-5p could upregulate the endogenous miR-125a-5p precursor expression in NSCLC cell lines (A549 and SK-MES-1), determined by qPCR. *n* = 3. *p < 0.05. (*d*) Successful over-expression of Suv39H1, determined by western blot in NSCLC cell lines (A549 and SK-MES-1). (*e*) Upregulation of endogenous miR-125a-5p precursor by exogenous miR-125a-5p over-expression could be abolished by Suv39H1 over-expression in NSCLC cell lines (A549 and SK-MES-1), determined by qPCR. *n* = 3. *p < 0.05. (*f*) The demethylation of miR-125a-5p by exogenous miR-125a-5p over-expression could be abolished by Suv39H1 over-expression in NSCLC cell lines (A549 and SK-MES-1). *n* = 3. *p < 0.05. NC: empty vector.

### 3.4. Over-expression of miR-125a-5p inhibits non-small-cell lung cancer activities

It has been demonstrated that miR-125a-5p functions as a tumour suppressor and our data also showed that its expression decreased in the NSCLC specimens. Thus, we further evaluated the anti-tumour effects of miR-125a-5p *in vitro*. Two NSCLC cell lines, A549 and SK-MES-1, were used. And our data showed that over-expressing miR-125a-5p could inhibit the cell migration (figure 4*a*; electronic supplementary material, figure S1), invasion (figure 4*b*) and proliferation (figure 4*c*) of NSCLC cells. In addition, the miR-125a-5p could accelerate the cell apoptosis of NSCLC cells (figure 4*d*).

**Figure 4.** Increasing miR-125a-5p level suppressed NSCLC cell activities. (*a*) Wound healing assay with over-expressing miR-125a-5p or empty vector (NC) in NSCLC cell lines (A549 and SK-MES-1). *n* = 3. *p < 0.05. (*b*) Cell invasion assay with over-expressing miR-125a-5p or empty vector (NC) in NSCLC cell lines (A549 and SK-MES-1). *n* = 3. *p < 0.05. (*c*) The survival rate analysis with over-expressing miR-125a-5p or empty vector (NC) in NSCLC cell lines (A549 and SK-MES-1). *n* = 3. *p < 0.05. (*d*) The cell apoptosis analysis with over-expressing miR-125a-5p or empty vector (NC) in NSCLC cell lines (A549 and SK-MES-1). *n* = 3. *p < 0.05.

### 3.5. Over-expressing miR-125a-5p suppresses non-small-cell lung cancer development *in vivo*

To further confirm the important role of miR-125a-5p level on NSCLC development, human NSCLC cancer cell line A549 was first infected with lentivirus expressing miR-125a-5p. Then the cells were transplanted subcutaneously into the dorsal scapula region of the nude mice. Data showed that over-expressing miR-125a-5p inhibited NSCLC development *in vivo* (figure 5*a*). Furthermore, exogenous miR-125a-5p over-expression could decrease the endogenous miR-125a-5p methylation level (figure 5*b*) and also promotes its precursor expression (figure 5*c*). The Suv39H1 level was also decreased after miR-125a-5p over-expression (figure 5*d*). These data showed that over-expressing miR-125a-5p inhibited NSCLC development *in vivo* through suppressing Suv39H1 expression, resulting in endogenous miR-125a-5p demethylation and upregulation.

**Figure 5.** Over-expressing miR-125a-5p suppressed NSCLC development *in vivo*. (*a*) Over-expressing miR-125a-5p decreased the tumour size *in vivo*. *n* = 12. *p < 0.05. (i) Statistical analysis; (ii) representative figures of the tumour formation. (*b*) Over-expressing miR-125a-5p decreased the methylation level of miR-125a-5p *in vivo*. *n* = 12. *p < 0.05. (*c*) Over-expressing miR-125a-5p increased the expression of endogenous miR-125a-5p precursor *in vivo*. *n* = 12. *p < 0.05. (*d*) Over-expressing miR-125a-5p suppressed the expression of Suv39H1 *in vivo*. *n* = 12. *p < 0.05. NC: empty vector.

## 4. Discussion

Lung cancer is one of the most common malignancies worldwide, and it remains the leading cause of cancer-related death, with low early-stage diagnosis rate. Owing to the complexity and heterogeneity of this disease, the early diagnosis of lung cancer can improve survival rate [19]. Therefore, more efforts should be made to uncover the underlying mechanisms and develop novel therapeutic targets.

miRNAs are a class of single-stranded non-coding RNAs that regulate target gene expression, predominantly by base pairing to the 3′-untranslated (3′-UTR) region of their target mRNAs [5–7]. Recent studies have established the presence of miRNA expression signatures in lung cancer, but our understanding of the function of aberrant miRNAs in lung cancer progression remains in its infancy [8–10]. miR-125a-5p has been previously reported to be downregulated in various human cancer types, including lung cancer [8–10]. Furthermore, miR-125a-5p has been validated to prevent the cancer cell progression [8–17,21,22]. However, the underlying mechanism of the low expression of miR-125a-5p in NSCLC remains unknown.

In the current study, it was further confirmed that miR-125a-5p expression was reduced in most NSCLC comparing with the adjacent non-tumour tissues. And the downregulation was tightly correlated with the low OS and DFS. DNA methylation analysis showed that the miR-125a-5p promoter was highly methylated and negatively associated its expression. Aberrant promoter methylation is considered a hallmark of cancer involved in silencing of tumour suppressor genes and activation of oncogenes. Aberrant DNA methylation includes hyper/hypomethylation. For tumour suppressor genes, such as miR-125a-5p, the molecules are commonly hypermethylated in tumour tissues compared with non-tumour tissues. In addition to our study here, miR-125a-5p has been demonstrated to be hypermethylated in glioma cells [25].

Target gene screening and validation showed that the histone methyltransferase Suv39H1 was the miR-125a-5p target gene that was also involved in the epigenetic silencing of the miR-125a-5p. It has been demonstrated that Suv39H1 is over-expressed in gastric cancers and knocking-down Suv39H1 could suppress gastric cancer development, which is in accordance with our results here [26]. In addition to the hypermethylation of the miR-125a-5p locus, other genetic and/or epigenetic events, such as HDACs and Sirtuins, might also participate into the miR-125a-5p repression [14,23,24]. Given previous work showing that SUV39H-mediated H3K9me3 controls DNA methylation in mammalian cells [27], it is highly likely that DNA hypermethylation of the miR-125a-5p locus is the downstream of SUV39H1 upregulation resulting from the miR-125a-5p repression. Furthermore, Suv39H1 is one of the known targets of miR-125b, which shares the same seed sequences with miR-125a [28]. Overexpressing miR-125a-5p could self-activate the silenced miR-125a-5p in NSCLC cells, resulting in cancer suppression *in vitro* and *in vivo*. The data here showed that miR-125a-5p might not only have the potential prognostic value as a tumour biomarker but also be potential therapeutic targets in NSCLC.

The identification of the expression levels and tumour suppressive function of miR-125a-5p in NSCLC provides a new window of therapeutic opportunity. The development of modified miRNAs with longer half-time and higher efficiency has produced favourable anti-cancer outcomes in experimental models, including locked nucleic acid modified oligonucleotides and antisense oligonucleotides [5–7]. Therefore, enforced expression of miR-125a-5p using approaches such as transfection of miR-125a-5p-carrying viruses or synthetic miR-125a-5p oligonucleotides will be required for future study in NSCLC therapies.

## Supplementary Material

Figure S1.

## Supplementary Material

Figure S2.

## Supplementary Material

Supplemental Table 1-Target prediction via miRDB.pdf

## Supplementary Material

Supplemental Table 2-Target prediction via TargetscanHuman 7.1.pdf

## Supplementary Material

Supplemental Table 3-Target prediction via PicTar.pdf

## Data accessibility

All data have been submitted as main figures or electronic supplementary figures.
